# Association between interleukin-21 gene rs6822844 polymorphism and rheumatoid arthritis susceptibility

**DOI:** 10.1042/BSR20190110

**Published:** 2019-08-15

**Authors:** Kewei Ren, Jilei Tang, Luming Nong, Nan Shen, Xiaolong Li

**Affiliations:** 1 Department of Orthopedics, The Affiliated Jiangyin Hospital of Southeast University Medical School, Jiangyin 214400, China; 2 Department of Orthopedics, Qidong People’s Hospital, Nantong 226200, China; 3 Department of Orthopedics, The Affiliated Changzhou No.2 People’s Hospital with Nanjing Medical University, Changzhou 213003, China; 4 Department of Clinical Pharmacy, The Affiliated Jiangyin Hospital of Southeast University Medical School, Jiangyin 214400, China; 5 Department of Orthopedics, The Affiliated Wujin Hospital of Jiangsu University, Changzhou 213002, China

**Keywords:** Interleukin-21, polymorphism, rheumatoid arthritis

## Abstract

Controversial results concerning the association between a polymorphism *rs6822844* in the interleukin (IL) 21 (IL-21) gene and rheumatoid arthritis (RA) have existed. A meta-analysis to confirm above relationships is necessary to be performed immediately. We conducted a search in the PubMed database, covering all papers published up to 20 October 2018. Overall, six case–control studies with 3244 cases and 3431 healthy controls were included. Odds ratios (ORs) and 95% confidence intervals (CIs) were used to assess the strength of this association. Publication bias was assessed with both Egger’s and Begg’s tests. After calculation, we found that *IL-21 rs6822844* polymorphism could decrease RA risk in overall genetic models (allelic contrast: OR = 0.77, 95% CI = 0.62–0.97, *P*=0.024; TG *versus* GG: OR = 0.68, 95% CI = 0.50–0.92, *P*=0.013, and dominant genetic model: OR = 0.72, 95% CI = 0.55–0.94, *P*=0.016). Similarly, stratified analysis by race, source of control, significantly decreased association was found in Asians, Caucasians and hospital-based (HB) control source. Finally, in the subgroup analysis of rheumatoid factor (RF) and anti-citrullinated protein antibody (ACPA) status, poorly decreased relationship was detected between *IL-21 rs6822844* polymorphism and RF negative and ACPA positive RA risk, respectively. No obvious evidence of publication bias was detected in overall analysis. In summary, our study indicated that *IL-21 rs6822844* polymorphism was significantly associated with decreased RA susceptibility.

## Introduction

Rheumatoid arthritis (RA) is a systemic, inflammatory autoimmune disorder with numerous manifestations caused due to intricate chain of events [1]. Cells of the leukocyte lineage such as: monocytes-macrophages, neutrophils, mastocytes, and subsets of T and B cells majorly contribute to the pathogenesis of RA by secreting various cytokines and chemokines [2].

Interleukin (IL) 21 (IL-21), a dual role cytokine discovered during the year 2000 shares similar homology with IL-2 family of cytokines (IL-2, IL-4, and IL-15) [3]. IL-21 interacts with γ chain (γc) of IL-21 receptor (IL-21R) expressed in various immune cells of the leukocyte lineage. IL-21 is predominantly secreted by T helper 17 (Th17) follicular T helper (Tfh) and natural killer T (NKT) cells [4].

In recent years, IL-21 has been found to be a key player in RA pathogenesis and progression [5–7]. In RA pathogenesis, IL-21R is highly expressed on CD4^+^ T-cell subsets, macrophages, dendritic cells, and synovial fibroblasts [8]. These immune cell subtypes recognize the IL-21 in the microenvironment to carry out several intricate chains of events [9]. IL-21 has been implicated to be an important target in RA therapy and several studies have been put forth to substantiate its role through activation of signaling pathways and in promoting inflammatory condition [10,11].

Several single-nucleotide polymorphisms (SNPs) situated in IL2/IL21 region including: *rs13151961, rs13119723, rs6840978*, and *rs6822844* have proven to be significantly associated with many autoimmune disorders, such as RA [12,13]. Of these, the *rs6822844* is a relatively common SNP, which locates in the intergenic region between IL21 and IL2 genes and shows the strongest association with RA susceptibility. There have been several studies testing this SNP for association with RA in Caucasian sample sets, with varying levels of supporting evidence (*P*=2.8 × 10^−4^ ∼ 0.24 × 10^−4^) [14–17].

Taking into consideration the extensive role of *IL-21 rs6822844* polymorphism in RA, hence, to derive a more precise estimation of the association of *rs6822844* polymorphism between IL-21 gene and RA risk, we performed a meta-analysis of all eligible case–control studies [15,16,18–21].

## Materials and methods

### Identification and eligibility of relevant studies

We conducted searches on the PubMed database, last search updated on 20 October 2018, with the keywords containing ‘IL-21’ or ‘interleukin 21’, ‘polymorphism’ or ‘variant’ and ‘rheumatoid arthritis’, without any restriction on language or publication year. Using these terms, a total of 16 articles were retrieved, of which 6 articles coincided with the inclusion criteria. We also screened references of the retrieved articles and review articles by a hand search.

### Inclusion criteria and exclusion criteria

Studies that were included in our analysis had to meet all the following criteria: (i) the study assessed the correlation between RA and *IL-21 rs6822844* polymorphism; (ii) case–control studies; (iii) sufficient genotype numbers for cases and controls. Accordingly, the following exclusion criteria were also used: (i) no control population; (ii) no available genotype frequency, and (iii) duplication of the previous publications.

### Data extraction

Two of the authors extracted all data independently, complied with the selection criteria. The following items were collected: first author’s last name, year of publication, country of origin, ethnicity, total case/control number, source of control, Hardy–Weinberg equilibrium (HWE) of controls, and genotyping methods.

### Statistical analysis

Odds ratio (OR) with 95% confidence interval (CI) was used to measure the strength of the association between *IL-21 rs6822844* polymorphism and RA based on the genotype frequencies in cases and controls. Subgroup analysis stratified by ethnicity was performed first. Source of control subgroup analysis was performed on two classifications: population-based (PB) and hospital-based (HB). Classification of RA based on rheumatoid factor (RF) subgroup analysis was performed: RF-positive (+) RA or RF-negative (−) RA; at the same time, the anti-citrullinated protein antibody (ACPA) subgroup was also assessed: ACPA-positive (+) RA or ACPA -negative (−) RA.

The fixed effects model and the random effects model were used to calculate the pooled OR. The statistical significance of the summary OR was determined with the *Z*-test. Heterogeneity assumption was evaluated with a chi-square-based *Q*-test among the studies. A *P*-value of more than 0.10 for the *Q*-test indicated a lack of heterogeneity among the studies. In case significant heterogeneity was detected, the random effects model (DerSimonian–Laird method) was used, however, the fixed effects model (Mantel–Haenszel method) was chosen [22,23]. For *IL-21 rs6822844*, we investigated the relationship between genetic variants and RA risk in allelic contrast (C-allele *versus* T-allele), homozygote comparison (CC *versus* TT), dominant genetic model (CC+CT *versus* TT), heterozygote comparison (CT *versus* TT), and recessive genetic model (CC *versus* CT+TT). Funnel plot asymmetry was assessed using Begg’s test and publication bias was assessed using Egger’s test [24]. The departure of frequencies of IL-21 gene polymorphism from expectation under HWE was assessed by χ^2^ test in controls using the Pearson chi-square test, *P*<0.05 was considered significant [25]. All statistical tests for this meta-analysis were performed with Stata software (version 11.0; StataCorp LP, College Station, TX).

## Results

### Eligible studies

In total, 16 articles were collected from the PubMed database via a literature search using different combinations of keywords. As shown in Figure 1, ten articles were excluded (other gene polymorphism, other kinds of disease, and some unrelative articles). Finally, six different articles were included in current meta-analysis, including 3244 cases and 3431 controls concerning the *IL-21 rs6822844* polymorphism and RA risk. All the RA patients were followed by the selection of individuals who fulfill the American College of Rheumatology (formerly the American Rheumatism Association) 1987 revised criteria for RA [26]. The controls were unrelated healthy, age, and ethnically matched individuals. Characteristics of studies of *IL-21 rs6822844* polymorphism are summarized in Tables 1 and 2. Finally, we checked the Minor Allele Frequency (MAF) reported for the five main worldwide populations in the 1000 Genomes Browser: East Asian (EAS), 0.001; European (EUR), 0.1531; African (AFR), 0.0113; American (AMR), 0.0605; and South Asian (SAS), 0.0685 (Figure 2). The MAF in our analysis was 0.1542 and 0.1790 in the case and control groups, respectively, both higher than the results in the EAS from 1000 Genomes Browser database.

**Figure 1:** A flowchart illustrating the search strategy used to identify association studies for *IL-21 rs6822844* polymorphism and RA risk

**Figure 2:** T-allele frequencies for the *IL-21* gene *rs6822844* polymorphism among cases/controls stratified by ethnicity Vertical line, T-allele frequency; Horizontal line, ethnicity type.

**Table 1:** Study characteristics from published studies on the association between *IL-21 rs6822844* polymorphism and RA risk

Author	Year	Country	Ethnicity	Case	Control	SOC	Case			Control				Genotype
							TT	TG	GG	TT	TG	GG	HWE	
Daha	2009	Netherlands	Caucasian	877	866	HB	116	53	708	126	73	667	<0.01	MALDI-TOF-MS
Maiti	2010	Turkey	Asian	354	368	HB	6	32	316	4	65	299	0.824	TaqMan
Louahchi	2016	Algeria	Asian	323	323	PB	6	31	286	10	80	233	0.336	TaqMan
Malinowski	2017	Poland	Caucasian	422	338	PB	6	103	313	4	79	255	0.438	TaqMan
Teixeira	2009	France	Caucasian	434	434	PB	8	99	327	11	110	313	0.719	TaqMan
Hollis-Moffatt	2010	New Zealand	Caucasian	834	1102	PB	30	221	583	29	330	743	0.285	TaqMan

Abbreviations: HWE, Hardy–Weinberg equilibrium of control group; MALDI-TOF-MS, polymerase chain reaction-matrix-assisted laser desorption/ionization time-of-flight mass spectrometry; PB, population-based; SOC, source of control.

**Table 2:** RA characteristics from published studies on the association for *IL-21 rs6822844* polymorphism

Author	Year	Ethnicity	Types	Case	Control	Case			Control		
						TT	TG	GG	TT	TG	GG
Louahchi	2016	African	ACPA−	73	323	9	9	55	10	80	233
Louahchi	2016	African	ACPA+	258	323	6	26	226	10	80	233
Louahchi	2016	African	RF−	101	323	1	7	93	10	80	233
Louahchi	2016	African	RF+	222	323	5	23	194	10	80	233
Daha	2009	Caucasian	ACPA-	228	866	8	60	160	126	73	667
Daha	2009	Caucasian	ACPA+	327	866	25	52	250	126	73	667
Daha	2009	Caucasian	RF−	250	866	20	38	192	126	73	667
Daha	2009	Caucasian	RF+	487	866	55	53	379	126	73	667

### Meta-analysis

In the overall analysis, significantly decreased association could be observed between RA risk and the variant genotypes of *IL-21 rs6822844* in three different genetic models from whole populations: in the allelic contrast (OR = 0.77, 95% CI = 0.62–0.97, *P*_heterogeneity_<0.001, *P*=0.024, Figure 3), the heterozygote comparison (OR = 0.68, 95% CI = 0.50–0.92, *P*_heterogeneity_<0.001, *P*=0.013) and the dominant model (OR = 0.72, 95% CI = 0.55–0.94, *P*_heterogeneity_<0.001, *P*=0.016) (Table 3).

**Figure 3:** Forest plot of RA risk associated with *IL-21 rs6822844* polymorphism (T-allele *versus* G-allele) in the overall analysis The squares and hori*z*ontal lines correspond to the study-specific OR and 95% CI. The area of the squares reflects the weight (inverse of the variance). The diamond represents the summary OR and 95% CI.

**Table 3:** Total and stratified subgroup analysis of *IL-21 rs6822844* polymorphism and RA risk

Variables	*n*	Case/Control	T-allele versus. G-allele			TG versus. GG			TT versus. GG			TT+TG versus. GG			TT versus. TG+GG		
			OR (95% CI)	*P_h_*	*P*	OR (95% CI)	*P_h_*	*P*	OR (95% CI)	*P_h_*	*P*	OR (95% CI)	*P_h_*	*P*	OR (95% CI)	*P_h_*	*P*
Total	6	3244/3431	0.77 (0.62–0.97)	<0.001	0.024	0.68 (0.50–0.92)	<0.001	0.013	0.92 (0.74**–**1.15)	0.487	0.465	0.72 (0.55–0.94)	<0.001	0.016	0.96 (0.77**–**1.20)	0.542	0.726
Ethnicity																	
Asian	2	677/691	0.48 (0.37–0.63)	0.115	<0.001	0.38 (0.28–0.53)	0.231	<0.001	0.74 (0.34**–**1.62)	0.202	0.456	0.42 (0.31–0.56)	0.148	<0.001	0.87 (0.40**–**1.89)	0.243	0.721
Caucasian	4	2567/2740	0.91 (0.82**–**1.01)	0.500	0.066	0.86 (0.75–0.99)	0.392	0.035	0.94 (0.75**–**1.18)	0.472	0.589	0.88 (0.78–0.99)	0.556	0.041	0.97 (0.77**–**1.22)	0.454	0.795
Source of control																	
HB	2	1231/1234	0.79 (0.68–0.93)	0.126	0.004	0.58 (0.44–0.78)	0.197	<0.001	0.89 (0.68**–**1.16)	0.459	0.378	0.67 (0.44**–**1.01)	0.083	0.059	0.92 (0.70**–**1.20)	0.398	0.528
PB	4	2013/2197	0.78 (0.55**–**1.10)	<0.001	0.160	0.73 (0.49**–**1.08)	<0.001	0.117	1.00 (0.68**–**1.48)	0.304	0.996	0.74 (0.50**–**1.10)	<0.001	0.133	1.06 (0.72**–**1.57)	0.401	0.761
RF status																	
RF+	2	709/1189	0.63 (0.32**–**1.24)	0.004	0.181	0.67 (0.19**–**2.43)	<0.001	0.544	0.75 (0.54**–**1.04)	0.673	0.085	0.61 (0.24**–**1.53)	0.001	0.292	0.75 (0.54**–**1.03)	0.950	0.074
RF−	2	351/1189	0.47 (0.15**–**1.46)	0.003	0.194	0.65 (0.08**–**5.44)	<0.001	0.689	0.52 (0.32–0.84)	0.466	0.008	0.49 (0.11**–**2.22)	<0.001	0.357	0.49 (0.31–0.80)	0.651	0.004
ACPA status																	
ACPA+	2	585/1189	0.60 (0.33**–**1.09)	0.010	0.096	0.80 (0.15**–**4.43)	<0.001	0.801	0.54 (0.36–0.82)	0.786	0.004	0.62 (0.23**–**1.72)	<0.001	0.362	0.52 (0.34–0.78)	0.454	0.002
ACPA−	2	301/1189	0.94 (0.75**–**1.20)	0.196	0.635	1.31 (0.18**–**9.33)	<0.001	0.786	0.99 (0.07**–**14.35)	<0.001	0.993	1.25 (0.94**–**1.66)	0.128	0.121	0.96 (0.05**–**20.27)	<0.001	0.977

Abbreviations: *P*_h_, value of *Q*-test for heterogeneity test; *P, Z*-test for the statistical significance of the OR.

In the subgroup analysis by ethnicity, there had been decreased relationships between RA risk and *IL-21 rs6822844* polymorphism in both Asians (T-allele *versus* G-allele: OR = 0.48, 95% CI = 0.37–0.63, *P*_heterogeneity_=0.115, *P*<0.001; TG *versus* GG: OR = 0.38, 95% CI = 0.28–0.53, *P*_heterogeneity_=0.231, *P*<0.001 and TT+TG *versus* GG: OR = 0.42, 95% CI = 0.31–0.56, *P*_heterogeneity_=0.148, *P*<0.001, Figure 4) and Caucasians (TG *versus* GG: OR = 0.86, 95% CI = 0.75–0.99, *P*_heterogeneity_=0.392, *P*=0.035 and TT+TG *versus* GG: OR = 0.88, 95% CI = 0.78–0.99, *P*_heterogeneity_=0.556, *P*=0.041, Figure 4 and Table 3). Similar results were also detected in HB subgroup (for example: TG *versus* GG: OR = 0.58, 95% CI = 0.44–0.78, *P*_heterogeneity_=0.197, *P*<0.001, Figure 5 and Table 3).

**Figure 4:** Forest plot of RA risk associated with *IL-21 rs6822844* polymorphism (TT+TG *versus* GG) in the ethnicity subgroup The squares and horizontal lines correspond to the study-specific OR and 95% CI. The area of the squares reflects the weight (inverse of the variance). The diamond represents the summary OR and 95% CI.

**Figure 5:** Forest plot of RA risk associated with *IL-21 rs6822844* polymorphism (TG *versus* GG) in the source of control The squares and horizontal lines correspond to the study-specific OR and 95% CI. The area of the squares reflects the weight (inverse of the variance). The diamond represents the summary OR and 95% CI.

In the stratified analysis by RF status, pooled associations were found between RF^−^ RA risk and *IL-21 rs6822844* polymorphism in the homozygote comparison (OR = 0.52, 95% CI = 0.32–0.84, *P*_heterogeneity_=0.466, *P*=0.008, Figure 6) and the recessive genetic model (OR = 0.49, 95% CI = 0.31–0.80, *P*_heterogeneity_=0.651, *P*=0.004) (Table 2).

**Figure 6:** Forest plot of RA risk associated with *IL-21 rs6822844* polymorphism (TT *versus* GG) in the autoantibody subgroup (RF and ACPA status) The squares and horizontal lines correspond to the study-specific OR and 95% CI. The area of the squares reflects the weight (inverse of the variance). The diamond represents the summary OR and 95% CI.

In the stratified analysis by ACPA status, pooled associations were found between ACPA+ RA risk and *IL-21 rs6822844* polymorphism in the homozygote comparison (OR = 0.54, 95% CI = 0.36–0.82, *P*_heterogeneity_=0.786, *P*=0.004, Figure 6) and the recessive genetic model (OR = 0.52, 95% CI = 0.34–0.78, *P*_heterogeneity_=0.454, *P*=0.002) (Table 2).

### Sensitivity analysis and publication bias

The Begg’s funnel plot and Egger’s test were performed to assess publication bias. The results did not suggest any evidence of publication bias (for example: T-allele *versus* G-allele, *t* = −1.6, *P*=0.184 for Egger’s test; *z* = 1.13, *P*=0.26 for Begg’s test) (Figures 7 and 8, and Table 4). Sensitivity analysis was performed to assess the influence of each individual study on the pooled OR by sequential removal of individual studies. The results suggested that no individual study significantly affected the overall OR dominantly (for example: T-allele *versus* G-allele, Figure 9).

**Figure 7:** Begg’s funnel plot for publication bias test (T-allele *versus* G-allele)

**Figure 8:** Egger’s publication bias plot (T-allele *versus* G-allele)

**Figure 9:** Sensitivity analysis between *IL-21 rs6822844* polymorphism and RA risk (T-allele *versus* G-allele)

**Table 4:** Publication bias tests (Begg’s funnel plot and Egger’s test for publication bias test) for *IL-21 rs6822844* polymorphism

Egger’s test						Begg’s test	
Genetic type	Coefficient	Standard error	*t*	*P-*value	95% CI of intercept	*z*	*P-*value
T-allele vs. G-allele	−3.837	2.394	−1.6	0.184	(−10.485, 2.810)	1.13	0.26
TG vs. GG	−3.972	2.067	−1.92	0.127	(−9.712, 1.768)	1.88	0.06
TT vs. GG	−0.452	0.564	−0.8	0.467	(−2.020, 1.114)	0.38	0.707
TT+TG vs. GG	−4.213	2.275	−1.85	0.138	(−10.531, 2.104)	1.13	0.26
TT vs. TG+GG	−0.453	0.565	−0.8	0.467	(−2.022, 1.115)	0.75	0.452

## Network of gene interaction of IL-21 gene

The network of gene–gene interaction for *IL-21* gene was utilized through String online server (http://string-db.org/) (Figure 10) [27].

**Figure 10:** Human IL-21 interactions network with other genes obtained from String server At least ten genes have been indicated to correlate with IL-21 gene. Abbreviations: IFNGR1, interferon γ receptor 1; IL2RA, IL 2 receptor, α; IL2RB, IL 2 receptor, β; IL2RG, IL 2 receptor, γ; IL4R, IL 4 receptor; IL6R, IL 6 receptor; IL7R, IL 7 receptor; IL12RB1, IL 12 receptor, β 1; IL21R, IL 21 receptor; IL23R, IL 23 receptor.

## Discussion

RA is a systemic autoimmune disease characterized by chronic persistent synovial joint inflammation resulting in bony erosion, cartilage loss, and often systemic disorders, such as subcutaneous rheumatoid nodules, secondary Sjogren’s syndrome, interstitial lung disease, and systemic vasculitis [28,29]. RA is considered as a complex condition in which a combination of risk alleles from different susceptibility genes predisposes to the development of the disease [30].

Among the different polymorphisms located in the IL2-IL21 region at 4q27, the *rs6822844 G/T* polymorphism was found to be the most significantly associated with autoimmune disease susceptibility, including RA [12,13]. To the best of our knowledge, *rs6822844* is in a noncoding polymorphism located between IL21 (upstream) and IL2 (downstream) with no molecular function identified. However, this polymorphism may play a role in autoimmunity by modulating the gene expression of these two genes or by being in linkage disequilibrium with a causative mutation. Interestingly, the neighboring sequences between up- and downstream for *rs6822844* show strong homology with mature microRNA [31,32]. MicroRNAs are post-transcriptional regulators that bind to complementary sequences in the 3′ UTR of target mRNAs, usually resulting in gene silencing inhibiting their translation [33]. The major allele G of the *IL2-IL21 rs6822844* polymorphism is conserved in all microRNA precursor hairpin structures. Therefore, it is possible that the mutation might abolish microRNA production, altering the expression of the genes regulated by this microRNA [34].

To indicate the relationship between *IL-21 rs6822844* polymorphism and RA risk, to the best of our knowledge, this was the first-time analysis to combine all the publications to evaluate above association. We performed a meta-analysis involving 3244 RA cases and 3431 controls. In overall analysis, decreased relationship was observed between *rs6822844* T-allele and RA risk. Furthermore, in the stratified analysis by ethnicity, we found that individuals who carried T-allele or TG genotype had decreased risk of RA both in Asians and Caucasians. Finally, the *rs6822844* polymorphism can decrease risk for ACPA^+^ or RF^−^ RA. This indicated *IL-21 rs6822844* T-allele was a protective factor for RA susceptibility.

In addition, we used the online analysis system String to predict potential and functional partners (Figure 10). Finally, ten genes were predicted. The highest score of association was IL-21R (Score = 0.996), however, IL-6R had the lowest scores (Score = 0.833). Tan et al. [35] employed RNA sequencing technology to explore the differentially expressed genes (DEGs) of RA patients compared with healthy volunteers. Combined DEGs and bioinformatics analysis indicated that the cytokine imbalance relevant to key molecules: extracellular signal-regulated kinase 1/2, p38 mitogen-activated protein kinase, tumor necrosis factor, colony-stimulating factor 3, IL-6 and interferon gene (IFNG) were responsible for the common comprehensive mechanism of RA [35]. van Steenbergen et al. [36] reported that *IL2RA-rs2104286* and soluble IL2Rα-level were associated with RA-persistence, which was known to act as a protective factor against multiple sclerosis, diabetes mellitus, and RA. Li et al. [37] indicated the *−590* site and *−174* site polymorphisms in the promoter of IL-4 and IL-6, respectively, may be associated with increased risk of RA and could be used as genetic markers for assessing the susceptibility and severity of RA. O’Doherty et al. [38] suggested that TT genotype in *IL-7 rs6897932* polymorphism was significantly associated with RA risk. Gomes da Silva et al. [39] suggested that the variants +*2199 A/C IL-23R* could contribute to RA development. Paradowska-Gorycka et al. [40] indicated that *IL-12p40* + *1188A/C* polymorphism and IL-12p70 protein levels may be associated with RA. Above information predicted IL family genes, such as IL2A, IL4, IL-6, IL-7, IL-23R, IL-12 and IFNG may influence IL-21 and regulate the RA development, which maybe become intervention and treatment target genes in the future. Besides, Do et al. [41] reported that IL-21 was dispensable for γδ T-cell IL-17A expression in lymph nodes, while Moser et al. [42] indicated that IL-21R signaling suppressed the IL-17A-producing γδ T-cell response in lung after influenza A virus infection. In addition, Huang et al. [43] suggested IL-21/IL-21R may act as a potent inhibitor of IL-17A-producing γδ T cells, controlling neutrophil-dependent inflammatory responses mediated by IL-17A-producing γδ T cells. From above we can see, IL-21 is a significant regulator for IL-17A.

Some limitations in our meta-analysis should be considered. Beginning, the number of published studies included in our meta-analysis remains not sufficiently large for a comprehensive analysis. Second, the interactions between gene–gene, gene–environment, and even different polymorphic loci of the same gene may modulate RA risk. Third, our meta-analysis was based on unadjusted estimates, while a more precise analysis should be conducted if individual data were available, which would allow for the adjustment by other covariates including age, sex, family history, environmental factors, disease stage, and lifestyle.

In summary, our present analysis showed the evidence that *IL-21 rs6822844* polymorphism was associated with significantly decreased RA risk not only in Asian but also in Caucasian populations and may be considered as a biomarker in the detection of susceptibility for RA. Therefore, further well-designed large studies, particularly referring to gene–gene and gene–environment interactions are warranted.

## Abbreviations

ACPA: anti-citrullinated protein antibody
CI: confidence interval
DEG: differentially expressed gene
EAS: East Asian
HB: hospital-based
IFNG: interferon gene
IL: interleukin
IL-21R: IL-21 receptor
MAF: minor allele frequency
OR: odds ratio
RA: rheumatoid arthritis
RF: rheumatoid factor
SNP: single-nucleotide polymorphism
